# BTXA regulates the epithelial–mesenchymal transition and autophagy of keloid fibroblasts via modulating miR-1587/miR-2392 targeted ZEB2

**DOI:** 10.1042/BSR20190679

**Published:** 2019-10-21

**Authors:** Zhanying Hou, Feixiang Fan, Po Liu

**Affiliations:** 1 Department of Dermatology, Shenzhen Longhua District Central Hospital, Shenzhen 518110, Guangdong, China; 2 Department of Burn and Plastic Surgery, Shenzhen Longhua District Central Hospital, Shenzhen 518110, Guangdong, China

**Keywords:** Autophagy, BTXA, Epithelial-mesenchymal transition, Keloid, miR-1587/miR-2392, ZEB2

## Abstract

Keloids are very resistant to treatment in dermatology and plastic surgical practice. The present study aimed to explore the underlying mechanism of botulinum toxin A (BTXA) treated human skin keloid fibroblasts (HSFBs) proving some new insights into keloids treatment. Expression of miR-1587 and miR-2392 were significantly down-regulated in keloid tissues and HSFBs, while the ZEB2 was a target of both and up-regulated in keloid tissues and HSFBs compared with the normal controls. BTXA could significantly increase the expression of miR-1587 and miR-2392 but decrease the expression of ZEB2. BTXA could significantly inhibit the proliferation, cell cycle, and migration and promote apoptosis and autophagy of HSFBs; however, miR-1587 and miR-2392 inhibitors could reverse these effects of BTXA on HSFBs. Silencing ZEB2 could significantly attenuate the effects of miR-1587 and miR-2392 inhibitors in promoting cell proliferation and migration and suppressing apoptosis and autophagy of HSFBs after treating with BTXA. BTXA could suppress the proliferation and migration and promote apoptosis and autophagy of HSFBs via modulating miR-1587/miR-2392 targeted ZEB2.

## Introduction

Keloid is a frequent disease in dermatology and plastic surgical practice and is characterized by pathologically excessive dermal fibrosis, accumulation of extracellular matrix, and infiltration of inflammatory cells [1,2]. Commonly, keloid often occurs in wound healing after burn treatment or trauma operation and affects more than 0.3–16% population worldwide [3]. Despite the development of medical technology, several methods have been explored for the treatment of keloids, such as surgical excision, corticosteroids, steroid, 5-fluorouracil injection, and radiation and pressure therapy [4]. However, the outcome of keloids treatment is still unsatisfied due to high recurrence rate [5]. Therefore, it is important to investigate the mechanism of fibroblasts in keloid to explore some new treatments for keloids.

In recent years, multiple researches have demonstrated that dysregulated proliferation and insufficient apoptosis of fibroblasts, which are the major component of keloids, are of importance progress during the development of keloids [6] and microRNAs (miRNAs) might play critical roles in these progressions. Liu et al. [7] have demonstrated that miR-21 could regulate the proliferation and apoptosis of keloid fibroblasts via modulating the expression of PTEN. Overexpression of miR-200b could significantly attenuate the proliferation but promote apoptosis of human hypertrophic scar fibroblasts [8]. In addition, miR-181a could regulate proliferation and apoptosis of keloid fibroblasts via targeting PHLPP2 in AKT signaling pathway [9]. Moreover, activating PI3K/AKT/mTOR pathway could enhance the sensitivity of keloid tissue to radiation damage via increasing apoptosis and reducing autophagy as well as NHEJ and HR repair pathway [10]. Moreover, epithelial-to-mesenchymal transition (EMT) of fibroblasts is also considered to contribute to the accumulation of collagen in keloid [11]. Besides, epigenetic alterations in keloid fibroblasts are also involved in the pathogenesis of keloids, such as DNA methylation, histone acetylation, and miRNAs dysregulation [12]. However, the associations between miRNAs and these regulatory mechanisms are still largely unknown.

Botulinum toxin A (BTXA) is a product of *Clostridium botulinum* and commonly used for focal dystonia, spasticity, and chronic migraine treatment [13]. Recent decade, BTXA has been recommended to ameliorate pathological scarring via inducing muscle relaxation and decreasing wound tension [4]. However, the detailed mechanism of BTXA in treating keloids is still largely unknown. A previous study revealed that BTXA treatment could significantly regulate the expression of TGF-β1, VEGF, and MMP1, indicating that BTXA might regulate the EMT progression to modulate the development of keloids [14]. However, the correlations and mechanisms between BTXA and miRNAs as well as its targeted genes, are still rarely reported.

Using miRNA microarray, miR-1857 and miR-2392 were identified to be significantly down-regulated in keloid tissues, indicating that they might play critical role in the etiology of keloids. To explore the detailed mechanism of miRNAs, expression of miR-1857, miR-2392, and ZEB2 were detected in clinical tissues and keloid-derived fibroblasts. In addition, the effects of BXTA on miR-1857 and miR-2392 in regulating cell behaviors of keloid-derived fibroblasts were also studies for further mechanism investigations. Specifically, the effects of BTXA on EMT-associated markers were also determined using Western blotting. With these investigations, we hope to provide some new reference for the clinical application of BTXA.

## Methods

### Clinical sample collection

The present study was authorized by the Ethic Committee of Shenzhen Longhua District Central Hospital (No. AF/SC-08/01.0) and all subjects had signed the informed consent files. This research has been carried out in accordance with the World Medical Association Declaration of Helsinki. Keloid tissue samples (*n*=16) and non-pathological scar adjacent normal skin tissue samples (*n*=8) were obtained from cesarean delivery patients at the Department of Dermatology, Shenzhen Longhua District Central Hospital. All patients were included as they were first diagnosed with keloids by histology examination and could not receive any treatment before surgical excision.

### Hematoxylin–Eosin and Masson’s staining

After collection, parts of tissues were fixed with 4% paraformaldehyde (PFA) at 4°C overnight. Then, tissues were dehydrated by gradient ethanol, permeabilized by xylene, and embedded with paraffin. Following this, tissues were cut into 4-μm slices and stained with Hematoxylin–Eosin (H&E) solution (Servicebio, Wuhan, Hubei, China) or Masson’s staining kit according to the manufacturers’ protocol. Finally, slices were mounted with neutral resins and analyzed by a light microscope (Nikon Eclipse 1000, Tokyo, Japan).

### Immunofluorescence

For tissue samples, paraffin tissue slices were dewaxed by heating and rehydrated with gradient ethanol. Then, EDTA antigen restore solution was used to repair antigens on slices in a microwave oven at the condition of moderate heat for 8 min, heat preservation for 8 min, and moderate-low heat for 7 min followed by natural cooling. Then slices were washed with PBS twice (3 min per time), blocked with 10% bovine serum albumin for 30 min, and incubated with ZEB2 (1:200, Abcam, Cambridge, MA, U.S.A.) at 4°C overnight. After washing with PBS for three times (3 min per time), slices were incubated with the secondary antibody (1:1000, Abcam, Cambridge, MA, U.S.A.) at room temperature for 50 min followed by DAPI staining at room temperature for 10 min. Finally, slices were washed with PBS for three times (5 min per time), mounted with anti-fluorescence quench sealing liquid.

For cell samples, cells were seeded on plates with a density of 1 × 10^4^ per well followed by grouping and transfection as aforementioned. Then, cells were harvested and seeded in slides in six-well plates at a density of 2 × 10^4^/200 μl per well. After 4-h cultivation at 37°C, 5% CO_2_, medium was discarded and 2 ml fresh medium was added overnight. On the second day, medium was removed, washed with PBS twice, and fixed with 4% PFA for 30 min at room temperature. Then, cell slides were washed with PBS triplicate (5 min per time) and incubated with 1 Ml Triton-X-100 for 20 min. After PBS triplicate washing (5 min per time), cell slides were incubated with primary E-cadherin (1:200, Abcam, Cambridge, MA, U.S.A.) or Vimentin (1:200, Abcam, Cambridge, MA, U.S.A.) antibody at 4°C overnight. Subsequently, with PBS triplicate washing (5 min per time), cell slides were incubated the secondary antibody (1:1000, Abcam, Cambridge, MA, U.S.A.) at 37°C for 2 h, washed with PBS for three times (5 min per time), and mounted with anti-fluorescence quench sealing liquid. Both tissue and cell samples were analyzed in an inverted florescence microscope (MOTIC AE2000, TED PELLA, Inc., Redding, CA, U.S.A.).

### Cell culture and transfection

Human skin keloid fibroblasts (HSFBs, BNCC342248), human normal skin fibroblasts (HSFs, BNCC338008), and 293T cells (BNCC100530) were purchased from the BeNa Culture Collection (Kunshang, Jiangsu, China) and maintained in Dulbecco’s modified Eagle’s medium (DMEM, Genview, Tallahassee, FL, U.S.A.) supplemented with 10% fetal bovine serum (FBS, Gibco, Grand Island, NY, U.S.A.) in a humidity incubator at 37°C with 5% CO_2_ at atmosphere. For transfection, miRNA inhibitor, mimic, siRNA, or negative control (NC) was transfected into cells using Lipofectamine 2000 (Invitrogen, Carlsbad, CA, U.S.A.) according to the manufacturer’s protocol. Sequences of miRNA inhibitor, mimic, siRNA, or NC were summarized in Table 1.

**Table 1:** Sequences for miRNA inhibitors, mimics, siRNA, or NC

Item	Sequences
NC	Sense: 5′-UUCUCCGAACGUGUCACGUTT-3′
	Antisense: 5′-ACGUGCCACGUUCGGAGAATT-3′
miR-1587 mimics	Sense: 5′-UUGGGCUGGGCUGGGUUGGG-3′
	Antisense: 5′-CAACCCAGCCCAGCCCAAUU-3′
miR-1587 inhibitors	Sense: 5′-CCCAACCCAGCCCAGCCCAA-3′
miR-2392 mimics	Sense: 5′-UAGGAUGGGGGUGAGAGGUG-3′
	Antisense: 5′-CCUCUCACCCCCAUCCUAUU-3′
miR-2392 inhibitors	Sense: 5′-CACCUCUCACCCCCAUCCUA-3′
siZEB2 (723-745)	Sense: 5′-GGACAGAUCAGCACCAAAUUU-3′
	Antisense: 5′-AUUUGGUGCUGAUCUGUCCUU-3′
siZEB2 (169-1591)	Sense: 5′-GGAGACAGAUCAGUAAUAUUU-3′
	Antisense: 5′-AUAUUACUGAUCUGUCUCCUU-3′
siZEB2 (3086-3108)	Sense: 5′-CCCUAUCAGUGUGAUAAAUUU-3′
	Antisense: 5′-AUUUAUCACACUGAUAGGGUU-3′

### Cell counting kit-8 assay

HSFBs were seeded in 96-well plates at a density of 8.0 × 10^3^ per well and cultured with complete DMEM overnight. Then, cells were transfected or treated with different concentrations of BTXA (Lanzhou Institute of Biological Products Co., Ltd, Gansu, China) for 24, 48, and 72 h. Then, 100 μl of Cell counting kit-8 (CCK-8) solution was added to each well and maintained for 1 h. Finally, the optical density (OD) value of each well at 450 nm was assessed.

### EdU assay

HSBFs were seeded in 48-well plates at a density of 2.0 × 10^4^ per well and cultured with DMEM overnight. Then, cells were transfected and treated with BTXA for 48 h. Following this, cells were harvested in a tube, incubated with EdU solution A at a final concentration of 50 μM for 2 h, washed with PBS twice, and fixed with 4% PFA at room temperature overnight. Subsequently, cells were washed with PBS twice and incubated with 0.5% Triton X-100 (in PBS) solution at room temperature for 10 min and washed with PBS for one time. Then, cells were resuspended in 1× Apollo staining solution, incubated at room temperature for 10 min, washed with 0.5% Triton X-100 (in PBS) solution for three times, and resuspended in PBS. Following this, cells were resuspended into 200 μl of 1× Hoechst 33342 solution and incubated for 30 min at room temperature. Finally, cells were washed with PBS twice and suspended into PBS for cell viability determination using a flow cytometry (BD, FACSCalibur, San Jose, CA, U.S.A.).

### Cell cycle and apoptosis analyses

Cell cycle and apoptosis of HSBFs were determined using flow cytometry. Briefly, HSBFs were seeded in a six-well plate followed by treatment for 48 h. Following this, HBSFs were were harvested, washed twice with cold PBS, and resuspended in 200 μl Annexin V/PI (MultiSciences, Hangzhou, Zhejiang, China) or PI for 15 min at dark at room temperature. Following this, cells were analyzed using flow cytometry (BD, FACSCalibur, San Jose, CA, U.S.A.).

### Wound healing assay

Cell migration was measured using wound healing assay. Briefly, HSBFs were seeded in a six-well plate followed by treatment and/or transfection. Then, a scar was scraped in cell monolayer by a tip. Following this, the medium was removed, washed with PBS triplicate, recorded by pictured, and maintained in DMEM without FBS for 48 h at 37°C. Finally, the scratch was pictured and analyzed by an inverted microscope (Motic, Wetzlar, Germany).

### Dual-luciferase reporter assay

Briefly, 293T cells were seeded in 48-well plates and maintained in 200 μl DMED with 10% FBS overnight. Following this, cells were transfected with miRNA mimic or/and plasmid psiCHECK2-wild-type (WT)/-mutant-type (MUT) using Lipofectamine 2000 (Invitrogen, Carlsbad, CA, U.S.A.) according to the manufacturer’s protocol. Vector psiCHECK2 was purchased from Promega (Beijing Biotech Co., Ltd, China). After transfection for 48 h, medium was discarded and cells were washed with PBS for three times and lysed with 100 μl passive lysis buffer (PLB) at room temperature for 15 min. Subsequently, 20 μl lysate was added to the luminescence test plate and light value was detected using the bioluminescence detector (Promega, GloMax, Madison, WI, U.S.A.) within 2 s. Following this, 100 μl LAR II solution was added to each sample and detected with 2 s. Finally, 100 μl of Stop & Glo Reagent was added to each well to terminate the reaction and light value was recorded within 2 s followed by analysis according to the manufacturer’s protocol.

### Transwell assay

HBSFs were seeded in a six-well plate overnight and transfected and/or treated with BTXA. Following this, cells were harvested, washed with PBS, and suspended in FBS-free DMEM containing 0.2% bovine serum albumin (BSA) at a density of 2 × 10^5^/ml. Subsequently, 100 μl cell suspension was mixed with 200 μl FBS-free DMEM and seeded in the upper chamber of transwell (Costor, New York, NY, U.S.A.). Meanwhile, 700 μl DMEM containing 10% FBS was added to the lower chamber of transwell. Following with 48 h culturing, medium in upper chamber of transwell was discarded, scraped with cotton swab to remove cells, and fixed with 4% PFA at room temperature for 20 min. Subsequently, transwell was stained with Crystal Violet solution at room temperature for 10 min. After washing with running water, membrane in the transwell was collected, mounted with neutral resins. Finally, successful migrated cells were analyzed by an upright microscope (OLYMPUS CX41, Tokyo, Japan) with six random views.

### Quantitative real-time PCR

TRIzol reagent (Takara, Dalian, Liaoning, China) was used to isolate total RNA from the cells and tissues. After qualifying using a Q6000 UV (Quawell Technology, San Jose, CA, U.S.A.), 2 μg of total RNA was reversed to cDNA using the Bestar qPCR RT Kit (DBI, Shanghai, China) according to manufacturer’s protocol. Following this, qPCR was performed on an ABI 7500 (Applied Biosystems, Foster City, CA, U.S.A.) using the SYBR Green Real-time PCR assay kit (DBI, Shanghai, China) with the following conditions: 95°C for 2 min and 40 cycles of 94°C for 20 s, 54°C for 20 s, and 72°C for 20 s. Primers of genes were designed as follows: ZEB2-forward, 5′-GCGATGGTCATGCAGTCAG-3′ and ZEB2-reverse, 5′-CAGGTGGCAGGTCATTTTCTT-3′; GAPDH-forward, 5′-TGTTCGTCATGGGTGTGAAC-3′ and GAPDH-reverse, 5′-ATGGCATGGACTGTGGTCAT-3′; miR-1875: 5′-CTCAACTGGTGTCGTGGAGTCGGCAATTCAGTTGAGCCCAACCC-3′, miR-2392: 5′-CTCAACTGGTGTCGTGGAGTCGGCAATTCAGTTGAGCACCTCTC-3′; and U6-forward: 5′-CTCGCTTCGGCAGCACA-3′ and U6-reverse: 5′-AACGCTTCACGAATTTGCGT-3′. Quantification of gene expression levels was analyzed using the 2^−ΔΔ*C*_t_^ method [15]. All samples were conducted in triplicate and average was calculated.

### Western blotting

Cells and tissues were lysed with RIPA lysis buffer (Beyotime, Shanghai, China) containing proteinase inhibitor cocktail (0.01%, Sigma, St. Louis, MO, U.S.A.). Then, the lysates were centrifuged at 4°C, 12000×***g*** for 10 min. Following this, the supernatants were harvested and concentration of protein solution was determined using BCA method (Prod, CA, U.S.A.). After this, 30 μg of protein was subjected to SDS/PAGE, transferred electrophoretically on a PVDF membrane, and blocked with 5% BSA (Sangon Biotech, Shanghai, China) at room temperature for 1 h. Subsequently, membranes were incubated with specific primary antibodies (ZEB2, E-cadherin, vimentin, p62, LC3B, and GAPDH; Abcam, Cambridge, MA, U.S.A.) at 4°C overnight, respectively. After washing with TBST for three times, membranes were incubated with Goat anti-rabbit/mouse secondary antibodies (Boster, Wuhan, Hubei, China) at room temperature for 40 min. Finally, membranes were washed and visualized using ECL-detection system (PerkinElmer, Boston, MA, U.S.A.).

### Statistical analysis

In the current study, statistical analyses were performed using GraphPad Prism 7.0 (La Jolla, CA 92037, U.S.A.). All experiments in the present study were performed at least in triplicate. Data were presented with mean ± standard deviation (SD) and comparisons among groups were analyzed using Student’s *t* test or one-way analysis of variance (ANOVA) with Tukey’s post hoc tests. For all comparisons, *P*<0.05 was considered statistically significant.

## Results

### Abnormal expression of miR-1587, miR-2392, and ZEB2 in keloid tissue which presented reducing dermal papilla but increasing collagen in reticular dermis

Both H&E and Masson’s staining assays have revealed that dermal papilla are significantly reduced in dermis but collagen was obviously accumulated in reticular dermis compared with the normal control skin samples (Figure 1A). Immunofluorescence had revealed that ZEB2 were markedly higher expressed in keloid tissues than normal skin tissue (Figure 1B). Quantitative real-time PCR (RT-qPCR) analysis had detected that the expression levels of miR-1587 and miR-2392 were significantly down-regulated in keloid tissues, but ZEB2 expression level was significantly up-regulated in keloid tissues compared with the normal skin tissues (Figure 1C). Further exploration had found that both expression levels of miR-1587 and miR-2932 were negatively correlated with the expression of ZEB2 in keloid tissues (Figure 1D). These findings indicated that miRNA-1587, miR-2932, and ZEB2 might play critical roles in the development of keloid and there might be some correlation between miR-1587/miR-2932 and ZEB2.

**Figure 1:** Expression of miR-1587, miR-2392, and ZEB2 in keloid tissues characterized by reducing dermal papilla but increasing collagen in reticular dermis (**A**) H&E and Masson’s staining analyses of keloid tissues. (**B**) Protein expression of ZEB2 in keloids and normal skin tissues. (**C**) Relative expression of miR-1587, miR-2392, and ZEB2 mRNA in keloids and normal skin tissues. (**D**) Significant expression correlation between miR-1587 and ZEB2 (R = 0.708, *P*<0.01), and miR-2392 and ZEB2 (R = 0.574, *P*<0.05). **P<0.01 and ***P<0.001 compared with the NS group.

### BTXA inhibits proliferation and cell cycle in HSFB cells via up-regulating miR-1587 and miR-2392 but down-regulating ZEB2

To further confirm our hypothesis, the expression of miR-1587 and miR-2932 were also detected and found that expression of miR-1587 and miR-2932 was significantly decreased in HSFB cells compared with the HSF cells (*P*<0.001, Figure 2A). However, BTXA treatment could significantly up-regulate the expression levels of miR-1587 and miR-2932 with a dose-dependent manner in HSFBs (*P*<0.001, Figure 2B). Meanwhile, BTXA treatment could also decrease the expression of ZEB2 in both mRNA and protein levels in HSFBs (*P*<0.001, Figure 2B,C). Both EdU and CCK-8 assays had revealed that BTXA could significantly inhibit the proliferation of HSFBs in a dose-dependent manner (*P*<0.001, Figure 2D,E). So 0.4 U/ml of BTXA was chosen as the optimal treatment concentration for subsequent experiments. Furthermore, BTXA could also induce an obvious accumulation in G_0_/G_1_ phase but a reduction in S phase of HSFBs (*P*<0.01, Figure 2F,G). However, no significant difference was identified in the G_2_/M phase of HSFBs cell cycle. These findings suggested that BTXA might control the proliferation of HSFBs via regulating the expression of miR-1587, miR-2932, and ZEB2.

**Figure 2:** BTXA effects on expression levels of miR-1587, miR-2392, and ZBE2, cell proliferation and cell cycle of HSFBs (**A**) Expression of miR-1587 and miR-2392 in HSF and HSFBs. (**B**) Expression of miR-1587, miR-2392, and ZEB2 after treating with BTXA in HSFBs. (**C**) Protein expression of ZEB2 in HSFBs. (**D**) Cell proliferation ability of HSFBs. (**E**) Cell proliferation activity of HSFBs. (**F,G**) Cell cycle of HSFBs. **P<0.01 and ***P<0.001 compared with the Control group.

### BTXA increases apoptosis and autophagy but suppresses the migration of HSFBs via regulating expression of ZEB2, E-cadherin, vimentin, p62, and LC3B

Furthermore, the apoptosis and migration of HSFBs was also determined after treating with BTXA. The result presented that BTXA could significantly increase the apoptosis in HSFBs (*P*<0.001, Figure 3A). Moreover, BTXA also decreased the migration ability of HSFBs (*P*<0.001, Figure 3B). Western blotting had further detected that BTXA could obviously reduce the expression levels of ZEB2, vimentin, p62, and LC3B-I, but increase the expression levels of E-cadherin and LC3B-II (Figure 3C). Immunofluorescence assay had found that BTXA could also inhibit the expression of Vimentin but elevate the expression of E-cadherin, which are important markers for EMT progress, in HSFBs (Figure 3D). These evidences suggested that BTXA might suppress the keloid progression via inhibiting EMT and increasing apoptosis and autophagy of HSFBs.

**Figure 3:** BTXA modulates cell apoptosis and cell migration of HSFBs via regulating the expression of ZEB2, E-cadherin, vimentin, p62, and LC3B (**A**) Apoptosis of HSFBs after treating with BTXA. (**B**) Cell migration of HSFBs. (**C**) Expression of EMT and autophagy associated markers. (**D**) Expression of E-cadherin and vimentin in HSFBs treated by BTXA. **P<0.01 and ***P<0.001 compared with the Control group.

### ZEB2 is a direct target of miR-1587 and miR-2392

According to the above description, there might be a relationship between ZEB2 and miR-1587/miR-2392. Bioinformatics analysis had informed that both miR-1587 and miR-2392 have interaction sites with ZEB2 (Figure 4A). Luciferase reporter assay revealed that overexpression of miR-1587 mimics or miR-2392 mimics could significantly reduce the WT, but not MUT, reporter activity of ZEB2 compared with the NC group (*P*<0.01, Figure 4B,C). These findings indicated that ZEB2 was the direct target of miR-1587 and miR-2392.

**Figure 4:** ZEB2 is a target of miR-1587/miR-2392 (**A**) Binding sites of miR-1587 and miR-2392 on ZEB2. (**B,C**) Regulatory relationships between miR-1587/miR-2392 and ZEB2 confirmed by dual luciferase activity assay. **P<0.01, compared with the NC group.

### miR-1587 or miR-2392 inhibitors reverse the effects of BTXA on HSFBs behavior via modulating the expression of ZEB2, E-cadherin, vimentin, p62, and LC3B

As aforementioned, BTXA could significantly increase the expression of miR-1587 and miR-2932, but decrease the expression of ZEB2. However, overexpression of miR-1587 or miR-2392 inhibitor could significantly reverse the effect of BTXA; namely, decrease the expression levels of miR-1587 and miR-2392, but increase the expression of ZEB2 (*P*<0.001, Figure 5A). EdU assay also depicted that miR-1587 or miR-2392 inhibitor could obviously reverse the proliferation inhibition of HSFBs induced by BTXA (Figure 5B). Moreover, miR-1587 or miR-2392 inhibitor could obviously attenuate the apoptosis elevation and migration reduction in HSFBs induced by BTXA (*P*<0.001, Figure 5C,D). In addition, miR-1587 or miR-2392 inhibitor could also ameliorate the reduction in ZEB2, vimentin, p62, and LC3B-I and reverse the accumulation of E-cadherin and LC3B-II induced by BTXA (Figure 5E). These findings suggested that miR-1587 or miR-2392 inhibitor could reverse the effect of BTXA on the behaviors of HSFBs.

**Figure 5:** miR-1587/miR-2392 inhibitor reverses the effect of BTXA on cell behaviors of HSFBs (**A**) Expression of miR-1587, miR-2392, and ZEB2. (**B**) Cell proliferation of HSFBs. (**C**) Apoptosis of HSFBs. (**D**) Migration of HSFBs. (**E**) Expression of EMT and autophagy associated markers. ***P<0.001 compared with the BTXA group.

### Silencing ZEB2 reverses the effect of miR-1587 or miR-2392 inhibitor on HSFBs behaviors

To further explore biofunction of ZEB2, ZEB2 was knocked down in HSFBs. According to the results, siZEB2-1569 showed the best effect in reducing the expression of ZEB2 in both mRNA and protein levels (Figure 6A). Therefore, siZEB2-1569 was used in the following HSFBs behavior detections. EdU assay had revealed that miR-1587 or miR-2392 inhibitor could obviously reverse proliferation reduction in HSFBs induced by BTXA, but silencing ZEB2 could markedly reverse the effect of miR-1587 or miR-2392 inhibitor to enhance the effect of BTXA on proliferation of HSFBs (Figure 6B). Moreover, silencing ZEB2 also could significantly increase the apoptosis of HSFBs after treating with BTXA and miR-1587/miR-2392 inhibitor (*P*<0.01, Figure 6C). Further transwell assay presented that knocked down ZEB2 could significantly inhibit the migration of HSFBs after treating with BTXA and miR-1587/miR-2392 inhibitor (*P*<0.01, Figure 6D). In addition, Western blotting also revealed that silencing ZEB2 could significantly decrease the expression of vimentin, p62, and LC3B-I but increase the expression of E-cadherin and LC3B-II after treating with BTXA and miR-1587/miR-2392 inhibitor (Figure 6E). These findings indicated that BTXA might regulate the behavior of HSFBs via regulating miR-1587/miR-2392-targeted ZEB2.

**Figure 6:** Silencing ZEB2 reverses the effects of miR-1587/miR-2392 inhibitor in attenuating HSFBs’ behaviors after treating with BTXA (**A**) Confirmation of silencing ZEB2 in both mRNA and protein levels. **P<0.01 and ***P<0.001 compared with the NC group. (**B**) Cell proliferation of HSFBs. (**C**) Apoptosis of HSFBs. ***P<0.001, ^##^*P*<0.01. (**D**) Migration of HSFBs. ***P<0.001, ^###^*P*<0.001. (**E**) Expression of EMT and apoptosis associated markers.

## Discussion

BTXA is a neurotoxic protein and effective in the treatment of several disorders [16–18]. In recent decade, BTXA has been recommended to treat keloid and achieved promising results [19]. However, the molecular mechanism of BTXA in treating keloid remains unclear. Recently, miRNAs are reported to involve in the progression of keloids, such as miR-29a [20], miR-1244-5p [21], and miR-141-3p [22]. Considering these, the correlations between BTXA and miRNAs in treating keloids were explored in the present study and found that BTXA was identified to regulate the expression of miR-1587 and miR-2392, and their targeted ZEB2 in HSFBs. In addition, miR-1587/miR-2392 inhibitors could obviously attenuate the effect of BTXA in reducing HSFBs proliferation and EMT, and inducing apoptosis via modulating the expression of ZEB2. It can be concluded that BTXA might play critical roles in the inhibition of proliferation and EMT and promotion of apoptosis and autophagy of keloid fibroblasts via miR-1587/miR-2392 targeted ZEB2.

miR-1587 and miR-2392 are two miRNAs newly identified in recent years. Specifically, miR-1587 contains G-rich sequences and has a probability to form intramolecular G-quadruplexes [23]. Glioma-associated mesenchymal stem cells secreted miR-1587 via exosomes, targeting, and reducing the expression of NCOR1 to promote proliferation and colony formation and increase cells tumorigenicity of glioma stem cells [24]. A previous study also revealed that miR-2392 might be a potential serum biomarker for cervical squamous cell carcinoma at early stage [25]. Li et al. have demonstrated that miR-2392 is down-regulated in gastric cancer cells and overexpression of miR-2392 inhibits metastasis and EMT via targeting MAML3 and WHSC1 in gastric cancer [26]. However, there are still rarely reports focused on the mechanisms of miR-1587 and miR-2392 in the progression of keloids. In the current study, both miR-1587 and miR-2392 were significantly down-regulated in keloid tissue and HSFBs and play critical roles in regulating the proliferation, apoptosis, autophagy, and EMT of HSFBs. In addition, BTXA could significantly inhibit the proliferation and EMT of HSFBs but promote apoptosis and autophagy via increasing the expression of miR-1587 and miR-2392 in a dose-dependent manner, and miR-1587 and miR-2392 inhibitors could significantly reverse these effects. These evidences suggested that miR-1587 and miR-2392 might play inhibitive roles the pathology of keloids and BTXA could improve the expression of miR-1587 and miR-2392 to suppress the proliferation and EMT of HSFBs but promote apoptosis and autophagy of HSFBs.

ZEB2, a receptor of Meox2, plays crucial role during phenoconversion [27]. Previous study had reported that p53 modulates EMT via miRNA targeted ZEB1 and ZEB2 [28]. Down-regulating the expression of miR-200a promote tumor growth and EMT via targeting E-cadherin repressors ZEB1/ZEB2 in Wnt/β-catenin pathway [29]. Meanwhile, Wnt/β-catenin pathway has been considered as a novel mediator for fibrosis and activated β-catenin in dermal fibroblasts promotes fibrosis via regulating extrasellar matrix associated gene expressions [30,31]. In this study, ZEB2 was identified to be a target of miR-1587 and miR-2392 and significantly up-regulated in keloid tissues. BTXA could significantly down-regulate the expression of ZEB2 in fibroblasts. An *in vivo* assay revealed that BTXA could significantly inhibit collagen deposition in hypertrophic scar rat model [32]. Furthermore, miR-1587/miR-2392 inhibitor could obviously attenuate the effect of BTXA in inhibiting the proliferation and migration of HSFBs and promoting apoptosis and autophagy, while silencing ZEB2 was obviously reversed these effects of miR-1587/miR-2392 inhibitor on BTXA-treated HSFBs. These findings suggested that BTXA might inhibit the fibrosis of keloids via down-regulating ZEB2, but the exact mechanism of BTXA in treating keloids still required further explorations.

## Conclusion

In conclusion, miR-1587/miR-2392 played an inhibitive role in the progression of keloids, and ZEB2, which could be targeted by miR-1587/miR-2392, played a promotive role in the development of keloids. BTXA could significantly down-regulate the expression of ZEB2 via up-regulating the expression of miR-1587/miR-2392 to suppress the proliferation and EMT but increase cell apoptosis and autophagy of HSFBs, to attenuate the development of keloids.

## Availability of Data and Material

All data generated or analyzed during the present study are included in this published article.

## Abbreviations

BSA: bovine serum albumin
BTXA: botulinum toxin A
CCK-8: cell counting kit-8
DMEM: Dulbecco’s modified Eagle’s medium
EMT: epithelial-to-mesenchymal transition
FBS: fetal bovine serum
HR: hypoxia reperfusion
HSF: human normal skin fibroblast
HSFB: human skin keliod fibroblast
H&E: Hematoxylin and Eosin
miRNA: microRNA
NC: negative control
PFA: paraformaldehyde
